RETRACTED

# Comprehensive Evaluation of Government Economic Management Performance Based on Multidimensional Data Mining in Fuzzy Comprehensive Environment

**DOI:** 10.1155/2022/4265125

**Published:** 2022-09-22

**Authors:** Min Wang

**Affiliations:** School of Public Administration, Central China Normal University, Wuhan 430079, China

## Abstract

Economic, political, social, and military activities all fall under the umbrella of government duties. The modification and reinterpretation of economic functions are the primary focus of the innovation in government administration style under the wave of economic globalisation. The effectiveness of the government's economic administration determines the general level of public administration at the federal level. An essential issue of national public administration that has a significant impact on the political growth of many nations is the performance evaluation of government economic administration. The people are the subject of government economic administration performance evaluation, and the people adjudicate the outcomes. An essential method of assessing the productivity of various departments is through performance review. The nation is currently in the process of switching from its long-standing planned economic system to a market economic system. The internal and external environments of governmental organisations are continually changing in addition to the strong trend of economic globalisation. Determining and advancing the national government's economic administration model is so crucial. The article offers a multidimensional data mining-based optimum design scheme for the thorough assessment of government economic administration performance. The fuzzy comprehensive evaluation rule is an effective method for quantifying the qualitative indicators when the quantitative indicators in the evaluation index system are difficult to measure. It is relatively simple, reasonable, and simple to operate in practise, which is conducive to the thorough and scientific performance evaluation of the government economic administration's science and technology administration functions. Following an assessment of the system's performance using association rule data mining technologies, a simulation test analysis is completed. The accuracy of the proposed arithmetic, which is 8.26% higher than the conventional arithmetic, is demonstrated by simulation results. The development of an evaluation model that incorporates both subjective and objective criteria, as well as the thorough assessment of the effectiveness of government economic administration based on data mining technologies, has excellent application prospects and practical value.

RETRACTED

## 1. Introduction

The so-called performance of government economic administration refers to the results and achievements of the government in economic administration activities. Obviously, it is of great significance to study the performance of government economic administration [1]. First, by studying the government administration performance, we can objectively judge whether the government economic administration is successful. Second, provide the direction of the government's future actions and efforts. Performance has many aspects, and the importance of each aspect depends on the value orientation of society and the social preferences of the public. If the performance of one or several aspects is limited, in fact, it also stipulates the behavioral objectives of the government's economic administration in the future. Third, through the study of government economic administration performance, we should also solve the cost-effectiveness problem of government self operation [2]. As a special social organization in the commodity economy, the government also follows the general law of commodity economy, that is, the law of value, to some extent [3]. However, through analysis, we should also explain the particularity of the government as a social organization with specific services and behavioral functions, which is different from general economic units or organizations [4]. Under the condition of commodity economy, the government, as an organization member in the society, its activities also occupy and consume various social and economic resources. Only by occupying and consuming these social and economic resources, the government can operate normally, provide various administration services required by the society, and individuals in the government economic administration organization can have the material conditions and economic foundation to play the role of public servants.

For government economic activities, it is not suitable to use the cost-benefit analysis way, and it is best to use relevant economic indicators to analyze the resource occupation and use of government behavior. This is due to two factors: first, it is challenging to assess the economic behaviour performance of government economic administration with precise costs and concepts; second, due to the phenomenon of administration time lag, the performance of its economic behaviour should not be clearly seen in a short period of time. With the advancement of database and artificial intelligence technology [5–7], data mining is a branch of information technology [8]. Data mining is a sophisticated processing technique used to extract from data sets useful, unique, potentially practical, and ultimately intelligible patterns. Data cleansing, data integration, data selection, data transformation, data mining, pattern evaluation, knowledge representation, and other steps are typically included in the KDD process. Data mining is one of them, and it forms the basis of KDD. The pattern to be discovered during the data mining operation is specified using the data mining function. Generally, the tasks of data mining can be classified into two categories: description and prediction. While the goal of predictive data mining is to deduce conclusions based on the most recent data for analysis and prediction, the goal of descriptive data mining is to characterise the overall properties of data in the database. Data mining technology has advanced significantly. The primary benefit of this approach is that it is not constrained by the amount of data and does not rely on past information. No matter how large the information and data are, objective data mining may always be done to uncover the underlying laws. The paper uses association rules and fuzzy comprehensive assessment in data mining to lower the execution cost of the math due to the benefits of this technology. Practice has shown that this combination can optimise government economic administration performance evaluation while also reducing computation time and enhancing evaluation quality and efficiency.

RETRACTED

In the process of national economic reform, the concept of cost has been brought into play to an unlimited extent [9]. When it comes to any reform measures, people will be referred to a problem of reform cost [10]. If there is also a cost problem in government behavior, it is mainly understood from a qualitative perspective, in addition to observing and accounting from the input-output perspective of a specific government organization, so it is not appropriate to extend it indiscriminately [11]. A reasonable approach is to draw conclusions about the cost of government economic administration and the performance evaluation of economic behavior through the realization of its behavior goals and the necessary quantitative analysis. Under the tide of economic globalization, the functions of the government should be changed, unchanged, and expanded. Without the targeted performance of the essential functions of the government, it is impossible to be fully prepared to meet the challenges of globalization. Therefore, the research on the functions of the government under the new economic conditions can enable the government to have a definite aim and concentrate on completing the affairs that most need the government's efforts. Article establishes a feature reconstruction model for the optimization design of the comprehensive evaluation of government economic administration, finds the optimal evaluation index of the government economic administration performance evaluation system through the fuzzy comprehensive evaluation way, extracts the relevant fuzzy feature quantity, and uses association rule data mining to test the optimization performance of the evaluation index. Its innovation lies in the following:

1. article adopts the way of association rules in data mining combined with fuzzy comprehensive evaluation in order to reduce the execution cost of the arithmetic
2. article constructs the key characteristic quantity of the optimal design of the evaluation of government economic administration, and adopts the way of comparing various arithmetics to realize the optimal design and optimal identification of the comprehensive evaluation of government economic administration

RETRACTED

## 2. Related Work

Government performance evaluation has a profound social background, which is directly driven by the decline of citizens' trust in the government [12]. When paying taxes, the public has the right to know the flow of taxes and fees. At the same time, the public is the recipient of public services, and also has information resources and qualifications to evaluate public services. Therefore, scientific and reasonable government performance evaluation is imminent.

Although the indicators of government performance evaluation are made up of several types, Kalkhoran et al. proposed that the primary performance indicators include output, efficiency, productivity, service quality, effect, cost-effectiveness, and customer satisfaction [13]. Jezeer et al. used Oregon as an example, discussed its government performance evaluation system, and introduced the Oregon government performance evaluation system, which had a total of 158 specific indicators in seven fields, including the economy, education, environment, citizen participation, social support, public safety, and community development [14]. The National Performance Evaluation Committee of the United States proposed the Government Performance Evaluation Index System, which is a set of evaluation indices including input, output, energy, result, efficiency, and cost-effectiveness, as well as productivity, and is subdivided into 150 to 1500 kinds [15]. Cowan and Schwab introduced the system. Vasev believes that there are many forms of government performance evaluation, such as evaluating input, evaluating output, or evaluating quality. When measuring the labor productivity of the government, people take the output of each person in a unit hour as a common index. These evaluation forms have their own purposes, and sometimes one or two of them can be used to complete an evaluation [16]. Taking the United States as an example, Cantador I and others introduced the representative government performance evaluation index system, including the evaluation model of the U.S. government accounting standards board, the evaluation model of the Campbell Institute, the general performance indicators of the federal government and the Balanced Scorecard evaluation model, and summarized the main experience and Enlightenment of the U.S. government performance evaluation [17]. Sun et al. introduced the contemporary federal government performance evaluation tools to evaluate federal projects; Department performance evaluation: federal departments evaluate department performance at the end of each fiscal year; The cross department performance evaluation mainly evaluates the progress of the federal departments in implementing the five reform plans in the presidential administration log through the three color rating bisection card [18]. Based on the logical model analysis, Dagaeva et al. pointed out that there is an obvious causal path in the whole process of government organizations from obtaining resources to output, and each key point on the path may be called a performance evaluation index. Different nodes correspond to three performance dimensions: stakeholder satisfaction, key issue resolution, and organizational administration status. The separate, pairwise combination and three-dimensional integration of different dimensions include the possible combinations of government performance evaluation [19]. Hong et al. divided the indicator system into three levels: the first level indicator evaluation dimension, the second level indicator focuses on the results of internal functions of the organization, and the third level can be divided into factor indicators, evidence indicators and quantitative indicators. In terms of design ways, different ideas such as key indicators, benchmarking administration, and factor relationships can be adopted according to the structure of performance elements [20]. Vandenrosch believes that the construction of local government performance evaluation index system is a systematic process, including five basic links: analysis of influencing factors of local government performance, analysis of performance evaluation characteristics, decomposition of performance evaluation objectives, screening and evaluation of performance evaluation indicators, and determination of index weight [21]. Zeng et al. proposed a three-dimensional logical framework for the design of performance evaluation index system based on “performance dimension-hierarchical characteristics sample attribute”, which can reflect all the information of the sample government performance in the performance range, specify the macro focus of the sample government performance in the spatial level, and reflect the historical basis and future development potential of the sample government in the sample attribute [22].

RETRACTED

Government performance evaluation is in the lead-in period; the theoretical ways are not mature, and the generally recognized research paradigm and system have yet to be formed. There are few research results on applicability and technical ways, emphasizing normative research over empirical research and general theoretical research, which have not yet gone deep into specific fields such as specific government levels, specific government departments, specific government projects, and so on. The article suggests a research and optimization design for a thorough assessment of the effectiveness of government economic administration based on multidimensional data mining. The comprehensive evaluation index of government economic administration is methodically constructed in this article using association rules in data mining technology and the fuzzy comprehensive evaluation method. The article then determines the optimal index, optimises the evaluation system, and optimises the distribution of government resources such as personnel, economic indicators, and other areas, making the operation of the comprehensive evaluation system more logical.

## 3. Methodology

### 3.1. Data Mining of Association Rules for the Analysis of Government Economic Administration Performance

The economic administration performance of government organizations cannot be measured by whether the activities of government organizations are profitable [23]. Society needs government organizations, not based on the idea of one more competing business competitor or partner, but on the desire to safeguard the environment and conditions of social and economic development and the interests of the public [24].

The multistage model regards the data discovery in the database as a multistage processing process, which includes many processing stages in the whole process of knowledge discovery.  Figure 1 is a simple diagram of the data processing model.

Data preparation, data mining, and pattern interpretation are the three processing phases that make up the KDD processing process in the processing paradigm shown in Figure 1. (1) Data preparation: comprehend the pertinent situation of KDD-related fields, including the preevaluation and application aims; be knowledgeable of the pertinent background assessment; be aware of the regulatory requirements. (2) Data mining: using the chosen data discovery mathematics, find or create a certain pattern or data set of interest, and then draw conclusions about the government's performance from the data. These assessments may be conveyed specifically or generally, for example, through production norms. (3) The following is the work's mode interpretation and evaluation's content: explain the found mode, get rid of the extraneous, irrelevant modes, and turn it into a constructive mode for assessment.

RETRACTED

A rules-based machine learning method called association rule mining can find relevant links in huge databases. Its goal is to use metrics to distinguish between the database's strong rules. Association rule mining is an unsupervised machine learning method since it is used for information discovery rather than prediction, discovering data patterns hidden in big data, mining association rules in potentially huge amounts of data, and increasing the efficacy of government economic administration performance evaluation. The performance assessment of government economic administration based on data mining technology is studied in this article, which also uses data mining technology to carry out data collection and analysis as well as performance assessment of government economic administration based on analysis outcomes. The important data regarding the effectiveness of the government's economic administration are mined using the association rule method, and the evaluation based on the mining results is carried out using the fuzzy comprehensive method. The example analysis findings demonstrate the great applicability of this method for assessing the performance of government economic administration.

Take the transaction data set as the object of association rule mining,

the binary text set is represented by *I* = {*i*_1_, *i*_2_, ⋯, *i*_*k*_}, and the elements in the set are called items. The item, that is, the set of transaction *T*, is represented by *D*, and needs to meet *T*⊆*I*. The unique identification of each transaction is represented by TID, and the set of items contained in *I* is represented by *X*. When *X*⊆*T*, it means that *X* is included in transaction *T*.

The implication form of association rules is *X*⇒*Y*, and there are *X* ⊂ *I*, *Y* ⊂ *I*, *X*∩*Y* = *φ*. The confidence, support, and correlation are used as the measurement indicators of association rules, and the values between 0% and 100% are used as the numerical interval of confidence and support.

The support and confidence of association rule *X*⇒*Y* are represented by *s* and *α*, respectively, which refer to the proportion of tuples *X* ∪ *Y* in transaction set *D* and the ratio of tuples *X* ∪ *Y* to *X* in transaction set *D*. The expression formula of support and confidence probability theory is as follows:

(1) $$\begin{array}{c} s\left(X\cup Y\right)=\mathrm{Pr}\left(X\cup Y\right),\\ \alpha \left(X\cup Y\right)=\mathrm{Pr}\left(X\cup Y\right)/\mathrm{Pr}\left(X\right). \end{array}$$

The degree of correlation refers to the degree of correlation between *X* and *Y*, and its probability theory expression formula is as follows:

(2) $$\begin{array}{c} \sigma_{X,Y}=\left\{\mathrm{Pr}\left(X\cup Y\right)\right\}/\left\{\mathrm{Pr}\left(X\right)\mathrm{Pr}\left(Y\right)\right\}. \end{array}$$

When *Pr*(*X* ∪ *Y*) = *Pr*(*X*)*Pr*(*Y*), *X* and *Y* are independent of each other.

RETRACTED

When the obtained correlation is greater than 1 and less than 1, it means that *X* and *Y* are positive correlation, and *X* and *Y* are negative correlation, respectively. When the association rule is negatively correlated, it means that the odds of the antecedent and the consequent are mutually inverse. The association rule needs to be removed because the logic is now illogical.

When the number of items in the itemset is *k*, it is called *k* itemset. The itemset support is the quantity of transactions that contain itemsets. The itemset is a frequent itemset if the minimal support is met. Assume that there is a transaction set *D* and that the association rules to be mined are the support and confidence rules that are greater than the minimum support and minimal confidence. The following is the definition of association rules:

(3) $$\begin{array}{c} s\left(X\Rightarrow Y\right)\geq s_{\min},\\ \alpha \left(X\Rightarrow Y\right)\geq \alpha_{\min},\\ \sigma \left(X\Rightarrow Y\right)\geq \sigma_{\min}, \end{array}$$

where *s*_min_≻0, *α*_min_≻0, *σ*_min_≻1.

### 3.2. Optimization Design of Government Economic Administration Performance Based on Fuzzy Comprehensive Evaluation Way

In order to make the design of local government economic administration performance evaluation index system more scientific, special attention should be paid to the dimension of public satisfaction survey. When establishing the public satisfaction evaluation index, the principles that must be followed are: (1) the established public satisfaction evaluation index system must be the most important to the public. Therefore, the primary problem is to accurately grasp the needs of the public and select the most critical evaluation indicators, such as social security and public safety; (2) The evaluation index must be measurable. As the public satisfaction survey is a quantitative value, the set evaluation indicators must be statistical, analytical, and calculable; (3) The evaluation index must be controllable. Public satisfaction evaluation will make the public have new expectations. It is feasible to adopt some ways to improve the performance evaluation index system of government economic administration and make it more scientific. For example, we can learn from the balanced scorecard way used in the performance evaluation of western government economic administration. The balanced scorecard is an index system of performance evaluation. Its core idea includes four indicators: finance, customers, internal business process, learning and growth, as shown in Figure 2.

RETRACTED

The data mining method of association rules is used to get the government economic administration performance assessment system, and the fuzzy comprehensive evaluation method is used to carry out the performance evaluation of public administration departments. The data mining-based performance review process used by the government economic administration is described as follows:

1. Define the evaluation index set. Set the index set *F* = {*F*_1_, *F*_2_, ⋯, *F*_*m*_} of the government economic administration performance evaluation system to include the evaluation index level as *F*; set the existing index set *S*_*i*_ = {*S*_*i*1_, *S*_*i*2_, ⋯, *S*_*im*_} as the evaluation factor set corresponding to *F*_*i*_
2. Establish judgment matrix. According to the evaluation index, the judgment matrix is established as follows:

(4) $$\begin{array}{c} P\left(F_{ij}\right)=\left[\begin{array}{c} F_{11},F_{12},\cdots ,F_{1m}\\ F_{21},F_{22},\cdots ,F_{2m}\\ .\cdots \cdots \cdots \cdots \cdots \cdots \cdots \\ F_{m1},F_{m2},\cdots ,F_{mm} \end{array}\right], \end{array}$$

where *F*_*ij*_ is the relative importance of index *F*_*i*_ to index *F*_*j*_, which is obtained according to Table 1.

(3) Calculate the weight. The formula of each column element in the normalized judgment matrix is as follows:

(5) $$\begin{array}{c} F_{ij}=F_{ij}/\overset{m}{\underset{k=1}{\sum }}F_{kj}, \end{array}$$

where *i*, *j* = 1, 2, ⋯, *m*.

Add the rows in the judgment matrix to obtain the normalization formula of each column of the judgment matrix as follows:

(6) $$\begin{array}{c} W_{i}=\overset{m}{\underset{j=1}{\sum }}F_{ij}. \end{array}$$

The *W*_*i*_ = *W*_*i*_/∑_*j*=1_^*m*^*W*_*j*_ way is used to normalize each index necklace, and the obtained result *W* = {*W*_1_, *W*_2_, ⋯, *W*_*m*_} is the weight vector.

(4) Fuzzy comprehensive. The “fuzzy set” is used as a mathematical model for describing fuzzy objects because it is based on the idea of precise mathematical sets and takes into consideration how the concept of sets has been modified and generalised. And gradually establish operation and transformation laws on the “fuzzy set,” and conduct pertinent theoretical research, it is possible to construct a mathematical foundation for studying a large number of fuzzy in the real world, and a mathematical way that can quantitatively describe and process fuzzy systems that appear to be quite complex. The scoring standard for each evaluation index must be established after the weights of each index in the index system have been determined. The scoring standard is determined using the fuzzy mathematics five point scoring method, and a fuzzy comprehensive evaluation model is then built. Use *X* = {*X*_1_, *X*_2_, ⋯, *X*_*i*_} to represent the factor set, *U* = {*U*_1_, *U*_2_, ⋯, *U*_*m*_} to represent the index set, *V* = {*V*_1_, *V*_2_, ⋯, *V*_*m*_} to represent the comment set, and establish the fuzzy transformation matrix *R*(*r*_*ij*_)_*m*×*n*_ as follows:

(7) $$\begin{array}{c} R=\left[\begin{array}{c} r_{11},r_{12},\cdots ,r_{1n}\\ r_{21},r_{22},\cdots ,r_{2n}\\ .\cdots \cdots \cdots \cdots \cdots \cdots \cdots \\ r_{m1},r_{m2},\cdots ,r_{mn} \end{array}\right]. \end{array}$$

In the formula, *r*_*ij*_ is the membership degree of level *j* evaluation of index *i*, and its calculation formula is as follows:

(8) $$\begin{array}{c} r_{ij}=V_{ij}/\overset{m}{\underset{i=1}{\sum }}V_{i}K_{i}, \end{array}$$

where *V*_*ij*_ means that the number of level *j* comments is *i*.

RETRACTED

The formula for calculating the average evaluation value is as follows:

(9) $$\begin{array}{c} B=W•R. \end{array}$$

When *B*_*j*_ = 1, it is necessary to normalize the average value in *B*_*i*_ = *B*_*i*_/*B*_*j*_ rows to obtain a result of *B* = {*B*_1_, *B*_2_, ⋯, *B*_*m*_}.

The formula for calculating the final score of index *X*_*i*_ is as follows:

(10) $$\begin{array}{c} D=B•\left\{V_{1},V_{2},\cdots ,V_{n}\right\}. \end{array}$$

The final evaluation of government economic administration performance is achieved through Equation (10).

## 4. Result Analysis and Discussion

The economic strength of a country can determine the overall level of the country to a certain extent. With the process of the country becoming more and more international, it is very necessary to strengthen economic administration. It is necessary to realize reasonable planning for the use of national funds, catch the development of various fields in the country, and achieve the improvement of the overall level. Through the research on the comprehensive evaluation of the government's economic administration performance, the innovation of the government's economic administration mode can complete the challenges of gradually realizing an open economy, integrating with the international administration mode, improving the national market economic system, and promoting the good development of the national economy in the context of economic globalization.

RETRACTED

The article uses association rules in data mining to mine network data and obtain evaluation-related data. If the threshold of support and confidence is set too low, it is simple to take too long to mine and there are weak association rules; if the threshold of support and confidence is set too high, useful association rules will be lost in the process of mining the data. Prior to counting the mining accuracy of this approach under various support and confidence levels, it is important to establish the support and confidence threshold for the association rule data mining approach.  Figure 3 presents the statistical findings. When the confidence level is 80% and the support level is 60%, according to the experimental results in Figure 3, the data mining accuracy is maximum in this case and exceeds 99%. The performance assessment of government economic administration uses the data mining approach of large data mining technology association rules. The support is 60%, and confidence in the data mining method of establishing association rules is 80%.

Figure 4 shows the memory occupation under different data sets. The less the memory occupation, the better the performance of the data mining arithmetic. It is more suitable for mining real large data sets. From the situation in Figure 4, the mining arithmetic based on association rule mapping occupies less memory capacity, while the data mining arithmetic based on rough set theory and heterogeneous information network occupies more memory capacity. Therefore, the arithmetic proposed in article has greater advantages in the performance of mining data sets.

The performance administration of government economic administration is extremely important to the improvement of national public administration level. The formulation of scientific and reasonable performance evaluation ways of government economic administration is extremely important to improve the government administration team. Using the evaluation results to evaluate the performance of government economic administration can improve the administrative ability of the government and realize the benign progress of government economic administration.

In order to test the evaluation performance of this way applied to the government economic administration performance, the other two ways of data analysis are selected as the comparison way, and the evaluation time of different ways in different data volume is counted. The comparison results are shown in Figure 5. From the experimental results in Figure 5, it can be seen that when this way is used to evaluate the government's economic administration performance, the evaluation can still be completed quickly within 15 s when the amount of data is 15GB. The real-time evaluation of this way is significantly higher than the other two ways, which can be applied to the government's economic administration performance evaluation in the big data environment and has high practicability.

RETRACTED

In order to verify the multidimensional data mining arithmetic based on the correlation rule mapping proposed in article, the experimental simulation hardware platform is IBM's PC; the main frequency is 2.3GHz CPU; the operating system is Windows XP, and the memory is 4GB. The software simulation platform is MATLAB7.0, and random real data sets are prepared in the experiment, including 800 data sets such as government economic data sets, public evaluation data sets, and government administration data sets. There are two sets of arithmetics used as comparisons in the experiment; one is an analysis way of heterogeneous information network data mining, and the other is a data mining way based on rough set theory. The experiment is divided into three parts, including memory consumption under different data sets, arithmetic mining accuracy at different data sets, and arithmetic running time at different data sets.

Figure 6 shows the mining accuracy of the arithmetic under the number of different data sets, and the larger the number of data sets, the better the mining accuracy can be maintained, which indicates the effectiveness of the mining arithmetic in practical application. It can be seen from the situation in Figure 6 that the proposed arithmetic occupies a leading position in terms of mining accuracy, and in the case of 800 data sets, the mining accuracy reaches 98%, while the mining accuracy of heterogeneous information network data is only 88%, and the arithmetic of rough set theory is 80%, and from the perspective of the change of mining accuracy when the number of data sets is increasing, the mining accuracy of this arithmetic is less affected.

Figure 7 shows the running time of the arithmetic under different data sets. The running time of the arithmetic increases with the increase of the number of data sets used. When the number of data sets is 800, the running time of the arithmetic in article is 16.7 s; the running time of sun arithmetic is 19.7 s, and the running time of BAL arithmetic is 21.3 s. The shorter the running time, the better reflects the advantage of the arithmetic in computing power. It is also more suitable for mining real large-scale data sets.

## 5. Conclusion

Article proposes an optimized design scheme for the comprehensive evaluation of government economic administration performance based on multidimensional data mining. The fuzzy comprehensive evaluation rule is an effective method for quantifying the qualitative indicators when the quantitative indicators in the evaluation index system are difficult to measure. It is relatively simple, reasonable, and simple to operate in practise, which is conducive to the thorough and scientific performance evaluation of the government economic administration's science and technology administration functions. Following an assessment of the system's performance using association rule data mining technologies, a simulation test analysis is completed. The accuracy of the proposed arithmetic, which is 8.26% higher than the conventional arithmetic, is demonstrated by simulation results. This complete result demonstrates the high effectiveness of the experimental verification method for assessing the efficiency of government economic administration, making it simple for the government administration department to pinpoint flaws and develop improvement plans for indicators with low scores. The establishment of government economic administration performance evaluation index system should follow the principles of purpose, integrity, independence, and comparability, that is, the index system should be able to reflect the information expressed by the original data more completely; all indicators should be independent of each other and affect each other; it should fully reflect the objectives of the evaluation and be fair and comparable to each evaluation object. Article in the construction of the performance database, the fact table and dimension table selection is not very reasonable, for the intelligent generation way of data conversion rules, some of the more accurate arithmetics, the arithmetic operation is not very high; the display of the results of the mining arithmetic needs to be further improved, providing a more humane and more friendly human-computer interaction interface, which can be further optimized according to the characteristics of performance data.

RETRACTED

## Figures and Tables

**Figure 1:** Process of data discovery in database.

**Figure 2:** Application of balanced scorecard in government economic administration performance evaluation.

**Figure 3:** Mning accuracy with different support and confidence.

**Figure 4:** Memory usage under different data sets.

**Figure 5:** Comparison of evaluation time of different ways.

**Figure 6:** Arithmetic mining accuracy under different data sets.

**Figure 7:** Arithmetic running time under different data sets.

**Table 1:** Determining the matrix scale.

Scale	Meaning
0-2	*F*_*i*_ is very less important than *F*_*j*_
2-4	*F*_*i*_ is less important than *F*_*j*_
4-6	*F*_*i*_ is as important as *F*_*j*_
6-8	*F*_*i*_ is more important than *F*_*j*_
8-10	*F*_*i*_ is very important compared with *F*_*j*_

## Data Availability

The data used to support the findings of this study are available from the corresponding author upon request.
